The article "Healthcare Waste Segregation Practice and Associated Factors among Healthcare Professionals Working in Public and Private Hospitals, Dire Dawa, Eastern Ethiopia" was published in 2023. Journal: J Environ Public Health.

# Healthcare Waste Segregation Practice and Associated Factors among Healthcare Professionals Working in Public and Private Hospitals, Dire Dawa, Eastern Ethiopia

**DOI:** 10.1155/2023/8015856

**Published:** 2023-01-28

**Authors:** Muna Ibrahim, Mesfin Kebede, Bizatu Mengiste

**Affiliations:** ^1^Dire Dawa Regional Health Bureau, Dire Dawa, Ethiopia; ^2^Department of Public Health, College of Medicine and Health Sciences, Dire Dawa University, Dire Dawa, Ethiopia; ^3^Department of Public Heath, St. Paul Teaching Hospital, Addis Ababa, Ethiopia

## Abstract

**Background:**

The key to the effective management of healthcare wastes is the segregation of the waste at the point of generation; no matter what final strategy for the treatment and disposal of wastes is selected, it is critical that waste streams are separated.

**Objective:**

The aim of the study is to assess the practice of healthcare waste segregation and associated factors among healthcare workers at public and private hospitals in Dire Dawa, Eastern Ethiopia.

**Methods:**

An institution-based cross-sectional study was conducted among 280 healthcare workers from public and private hospitals. Data were collected through self-administered structured questionnaires and observation checklists. Bivariate and multivariable logistic regression were used to identify factors associated with the practice of healthcare workers using SPSS (Statistical Package for Social Sciences) version 25.

**Results:**

This study showed that 56.4% (95% CI: 43.7–60.2) study participants had good healthcare waste segregation practices. Working in a public hospital (AOR = 0.09, 95% CI: (0.03–0.23)), working less than 40 hours a week (AOR = 4.28, 95% CI: (2.11–8.68)), adequate knowledge on healthcare waste management (AOR = 2.42, 95% CI: (1.27–4.61)), ever trained on waste management ((AOR = 2.74, 95% CI: (1.15–6.53)), the presence of guidelines, instructive posters on healthcare waste segregation ((AOR = 8.21, 95% CI: (3.84–17.55)), and availability of color-coded waste bins ((AOR = 9.53, 95% CI: (4.52–20.10)) were factors significantly associated with healthcare waste segregation practices.

**Conclusion:**

The study revealed that healthcare waste segregation practices were unacceptably poor. It is very crucial to address the identified factors through ongoing enforcement of healthcare waste management rules and regulations, by providing training, instructive posters around the work area, and making color-coded bins available.

## 1. Background

Healthcare waste management is critical because medical waste is contagious and dangerous, and it can harm people and the environment. Healthcare wastes include all the waste generated by healthcare establishments as well as the waste produced during patients' care at home [1, 2]. Healthcare wastes contain pathogenic agents and therefore constitute a substantial portion of healthcare wastes, which are hygienically dangerous, and the remaining minority of wastes include sharps, genotoxic wastes, heavy metals, chemicals, and pharmaceuticals. Healthcare wastes represent most hazardous wastes from healthcare facilities [3, 4].

The article "Healthcare Waste Segregation Practice and Associated Factors among Healthcare Professionals Working in Public and Private Hospitals, Dire Dawa, Eastern Ethiopia" was published in 2023. Journal: J Environ Public Health.

Safe healthcare waste management procedures, which encompass all waste creation, segregation, transportation, storage, treatment, and disposal activities, represent the caliber of the services provided in any healthcare facilities [5]. Segregation of waste at the point of generation is essential for healthcare waste mitigation and management. Regardless of the ultimate approach chosen for the treatment and disposal of waste, it is crucial that waste streams be separated to protect both humans and the environment [6–8].

According to a 2009 World Health Organization (WHO) study, around 20% of wastes is considered hazardous wastes. However, studies revealed that the percentages of these wastes generated from healthcare settings exceeded the WHO threshold that was due to poor waste segregation practices at the point of generation [9–11]. This poses a significant risk to humans and the environment, including injuries, infection transmission, pollution, fire hazards, and public nuisances [3, 12].

Healthcare waste segregation is particularly important in minimizing the volume of hazardous waste by making it easy to assess the composition of generated waste. Improper HCW segregation can increase disposal costs and present several risks to the environment and public health [13]. WHO has reported that exposure to sharps in the workplace accounts for 40% of Hepatitis B and Hepatitis C virus and 2%-3% of HIV infections among healthcare workers worldwide [3]. Hence, healthcare workers and waste handlers are at a risk of acquiring these diseases because of improper practices related to HCWs segregation [1, 14, 15].

However, proper wastes segregation should produce a safe solid waste stream that can be managed through recycling, composting, and landfilling easily, safely, and affordably [12, 16]. Through rigorous item separation, the number of wastes in the entire HCWs stream could be decreased by as much as 60%. In Ethiopia, the proportion of the hazardous waste generation rate becomes unacceptably high, ranging from 21 to 75% [17]. This discrepancy in the proportion of hazardous waste generation rate may be due to poor segregation practices of the workers at the point of generation and weak regulatory or enforcement of healthcare waste management systems [15, 18–21]. It would be useful to develop an effective system of waste characterization in both public and private hospitals. This is particularly important in ascertain how resources are allocated in the management of healthcare waste [13, 22].

The article "Healthcare Waste Segregation Practice and Associated Factors among Healthcare Professionals Working in Public and Private Hospitals, Dire Dawa, Eastern Ethiopia" was published in 2023. Journal: J Environ Public Health.

Even though the rules and regulations are the same all over Ethiopia, healthcare waste has not gotten the attention it deserves and there is limited evidence, particularly on healthcare waste segregation practices among the workers [15, 17, 19, 23–26]. Therefore, to create treatments to enhance the waste management system, it is crucial to comprehend the fundamental causes of HCW segregation practices in this regard. This study endeavors to assess the gap in the practice of healthcare waste segregation and associated factors among healthcare workers in Dire Dawa, Eastern Ethiopia.

## 2. Methods and Materials

### 2.1. Study Area and Period

Dire Dawa is in the eastern part of the country, enclosed by the state of Somalia and the state of Oromia. It is found at 515 kilometers from Addis Ababa, and it lies at an altitude and longitude of 9036″N 41052″E. There are 9 urban and 38 rural administrations. According to the 2012 population projection, the study area has a population of 506,639, with 51% female and 49% male. Most of the people (68%) are urban dwellers and the rest (32%) are rural dwellers. The economy of the city depends on trade and industry [27]. The city administration has a total of 5 hospitals (2 public hospitals and 3 private hospitals). A study was conducted from October 01 to November 30, 2020, in hospitals in the city.

### 2.2. Study Design

An institution-based cross-sectional study was conducted.

### 2.3. Study and Source Population

The source population was all health professionals who were working in either private or public hospitals in Dire Dawa.

The study population was health professionals working in the randomly selected hospitals.

### 2.4. Inclusion and Exclusion Criteria

The inclusion criteria were as follows: all health professionals in the hospital who directly engaged in activities generating both general and hazardous wastes, including medical doctors, health officers, laboratory professionals, midwives, and nurses.

The exclusion criteria were as follows: health professionals who had work experience of less than 6 months, who were working for free service, or who were parttime workers.

### 2.5. Sample Size Determination

The sample size was determined using a single population proportion formula with the assumption of 95% confidence level, 5% precision, considering the proportion of healthcare workers who had good HCWs segregation practice was 53.8% in southeast Ethiopia hospitals (22), and considering a possible nonresponse rate of 10%. Finally, a correction formula for a finite population was applied using the total number of health professionals working in all hospitals in Dire Dawa (*N* = 1150) and the final sample size was 287.

The article "Healthcare Waste Segregation Practice and Associated Factors among Healthcare Professionals Working in Public and Private Hospitals, Dire Dawa, Eastern Ethiopia" was published in 2023. Journal: J Environ Public Health.

### 2.6. Sampling Procedure

Initially, two hospitals were randomly selected, representing public and private hospitals. Then, the total sample size is distributed proportionally to the number of health workers found in the selected hospitals. From each of the hospitals, stratified proportionate sampling was again employed to select the different professional categories of health workers. Finally, from each stratum, simple random sampling was used to select the study participants.

### 2.7. Data Collection Methods

Data were collected using a structured and pretested questionnaire, as well as an observational checklist developed based on related studies and in accordance with COVID-19 precautions. A self-administered questionnaire was used to collect the data. An observational checklist was used to assess the practice in terms of segregation, while the study subjects were doing their task; then, a self-administered questionnaire was given to the study subjects.

### 2.8. Operational Definition

HCW segregation practice was assessed by nine items (presence of puncture resistance safety box, on-site sharp waste segregation, position of the safety box, separate waste collection container, on-site segregation of infectious and noninfectious wastes, labeled waste collection container, color-coded waste containers, and waste containers with covers).

Knowledge on HCW segregation was measured using ten items; then, it was categorized using mean score. Those who scored above or equal to the mean were labeled “adequate” and “inadequate” for who scored below the mean [23].

Attitude toward HCW segregation variables comprised of 6 statements with response categories “agree,” “disagree,” or “neutral.” Composite scores were calculated and those scored equal to and above the mean value for the composite score of attitude questions were labeled as having “favorable attitude” toward HCWs segregation, if not “unfavorable attitude” [18].

### 2.9. Data Quality Control

The self-administered questionnaire and observation checklist were prepared in English and translated into local languages. The questionnaire was pretested to identify potential problem areas with any of the questions among 14 respondents having similar characteristics to the study subjects. Training of data collectors and supervisors and pretesting of the questionnaire were performed to ensure the quality of the data. Daily, the completeness and consistency of the information gathered were double-checked and reviewed.

The article "Healthcare Waste Segregation Practice and Associated Factors among Healthcare Professionals Working in Public and Private Hospitals, Dire Dawa, Eastern Ethiopia" was published in 2023. Journal: J Environ Public Health.

### 2.10. Data Analysis

Data were entered, coded, and cleaned using Epi Data Version 3 statistical software and then exported to SPSS version 25.0 for further analysis. Descriptive statistics were performed for variables in the study using two statistical parameters: mean and percentage. Bivariate and multiple logistic regression were used to identify factors associated with healthcare workers waste segregation practices using *p*-values <0.05 as the cutoff point.

### 2.11. Ethical Considerations

Ethical clearance was obtained from the Dire Dawa University Research Ethics Review Committee (RERC). Informed written consent was obtained from the hospital's Chief Executive Officer (CEO) and all subjects for their participation after the nature of the study was fully explained to them. A signature was used on the consent form. All study participants were informed that the data would remain private and confidential and would be used only for research purposes. The participants were assured that they had the right to refuse or withdraw if they were not comfortable at any time.

## 3. Result

### 3.1. Sociodemographic Characteristics

A total of 280 health professionals participated in the study with a response rate of 97.6%, and out of them, 228 (81.4%) and 52 (18.6%) professionals were working in public and private hospitals, respectively. The overall mean age of the respondents was 33.3 (6.65) years, and the majority (173 or 61.8%) of the participants were female. Out of the 280 majority, 200 (71.4%) were married and 250 (89.3%) were found to have a first degree. Regarding the professional category, more than half (65.7%) were nurses, and the mean working hours per week was 44.07 hours (±SD18.843) (See Table 1).

### 3.2. Institution-Related Characteristics

Out of 280 study participants, 191 (68.2%) were working less than or equal to 40 hours per week and the remaining 89 (31.8%) worked more than 40 hours per week. Approximately, 203 (72.5%) and 175 (62.5%) had ever been trained healthcare waste management in the last one year. Additionally, 181 (64.6%) health professionals had color-coded waste bins and safety boxes around their work area. About 166 (59.3%) knew the rules and regulations on HCWM. 157 (56.1%) and 144 (51.4%) reported that there are supervision and control measures regarding waste management in hospitals.

### 3.3. Behavior-Related Characteristics

Based on ten knowledge-related items, the knowledge of health workers on healthcare waste segregation practice was 224 (80%) (See Table 2). Regarding attitude toward healthcare waste segregation practice, 159 (56.78%) of the respondents had a positive attitude. Around 182 (65%) of participants were observed to wear appropriate personal protective equipment (PPE). About 40 (85.7%) of study participants reported using appropriate PPE.

The article "Healthcare Waste Segregation Practice and Associated Factors among Healthcare Professionals Working in Public and Private Hospitals, Dire Dawa, Eastern Ethiopia" was published in 2023. Journal: J Environ Public Health.

### 3.4. Healthcare Waste Segregation Practice

Based on nine practice-related items and a cut-off point of 5.503 SD 2.75, 158 (56.4%) (95% CI: 43.7–59.2) of the study participants reported good healthcare waste segregation practice. From the observation assessment, 181 (64.6%) of respondents segregated waste in the available color-coded bin, and the presence of guidelines, standard operating procedure (SOP), or instructive posters was observed; thus, 143 (51.1%) were observed to practice waste segregation appropriately.

### 3.5. Factors Associated with Healthcare Waste Segregation Practices

In multivariate logistic regression analysis, hospital ownership, weekly working hours, knowledge of HCWs segregation, training in HCWM, presence of guidelines, SOP, or instructive poster on HCW segregation, and availability of a color-coded waste bin in the work area were the factors significantly associated with HCWs segregation practice. Healthcare workers working in public hospitals were 91.2% less likely to have good practices in infectious waste segregation than respondents who were working in private hospitals.

Healthcare workers who had worked less than 40 hours weekly had four times (AOR = 4.28, 95% CI: (2.11–8.68)) higher odds of having good practice compared to their counterparts. Health professionals who had adequate knowledge of HCWs' segregation had approximately two times (AOR = 2.42, 95% CI: (1.27–4.61)) higher odds compared with those who had inadequate knowledge. The odds of being trained on HCWM were three times higher ((AOR = 2.74, 95% CI: (1.15–6.53)) among trained workers than among those who had not been trained in the previous 12 months.

Moreover, the presence of guidelines, SOPs, or instructive posters on HCW segregation ((AOR = 8.21, 95% CI: (3.84–17.55)) was higher compared to their counterparts. Those who had color-coded waste bins around their work area had approximately nine times ((AOR = 9.53, 95% CI: (4.52–20.10)) higher odds of having good practices than those who did not have them (See Table 3).

## 4. Discussion

The key to the effective management of healthcare wastes is the segregation of the waste at the point of generation; no matter what final strategy for the treatment and disposal of wastes is selected, it is critical that waste streams are separated. The study aimed to assess healthcare waste segregation practices and associated factors among health professionals in Dire Dawa hospitals. This study shows that 56.4% of healthcare professionals had good healthcare waste segregation practices; sorting general, infectious, and sharp waste in different color-coded bins/boxes. This is comparable with studies conducted in Southeast Ethiopia (53.8%), Northwest Ethiopia (46.3%), and Addis Ababa, Ethiopia (43.2%)[15, 18, 26]. This finding is unacceptably higher and might contribute to the generation of a huge volume of hazardous waste from hospitals that exceeds the WHO threshold [9–11]. These figures may differ between health facilities and countries for a variety of reasons.

The article "Healthcare Waste Segregation Practice and Associated Factors among Healthcare Professionals Working in Public and Private Hospitals, Dire Dawa, Eastern Ethiopia" was published in 2023. Journal: J Environ Public Health.

Health professionals working in public hospitals were 91.2% less likely to have good practices of healthcare waste segregation than private hospitals. In line with this, the study conducted in Addis Ababa also revealed that healthcare waste segregation practice was reported to be minimal in public health facilities [28]. This might be due to lack of availability of color-coded containers around work area, poor attention, and absence or nonexistent control measures on healthcare waste management.

Healthcare workers who had worked less than 40 hours a week had four times higher odds of having good practice compared with those who worked more than 40 hours a week. This study revealed that long working hours contribute to poor HCW segregation practices. This might be due to fatigue and lack of attention while workers carried out routine activities, and there could also be accident injuries and exposures from improperly sorted waste [3, 29].

Moreover, healthcare workers who had ever been trained on HCWM were more likely to have good practices in waste segregation. This is consistent with the previous studies conducted in Gondar town, Northwest Ethiopia [24] and Dawro zone, Southwest Ethiopia [30]. Similarly, those who had adequate knowledge were 2.4 times more likely to practice healthcare waste segregation practices. The study conducted in South Africa also suggested that there is a significant relationship between knowledge and practice [31]. Similar studies also suggested that this finding is similar to that of Malini and Eshwar, who reported a lack of awareness and knowledge among the staff about hospital waste management [32]. Thus, allocating adequate resources with good managerial commitment to conduct training and educate the staff on rules and regulations of healthcare waste management might enhance and maintain good practices.

The waste management policy or guideline is the managing rule of healthcare workers and health facilities [33]. This study revealed that presence of guidelines, SOPs, or instructive posters around the work area is more likely to encourage the workers to practice good HCW segregation. Providing instructive posters as a tool to promote effective segregation of healthcare waste appears to have a positive effect among healthcare workers.

The article "Healthcare Waste Segregation Practice and Associated Factors among Healthcare Professionals Working in Public and Private Hospitals, Dire Dawa, Eastern Ethiopia" was published in 2023. Journal: J Environ Public Health.

Proper placing of waste in the ward with appropriate containers requires the assurance of adequate materials for collection of healthcare waste [21]. Those health professionals who have color-coded waste bins in their work area were 9.5 times more likely to practice than their counterparts. This finding is similar to the findings from Gonder town and Debree Markos hospitals [23, 25]. In general, as suggested by [34], enhancing awareness of 6 HCWM to healthcare staff and availing appropriate waste management utilities and enforcement from the regulatory bodies might improve the existing poor practices.

The strength of this study was that both public and private facilities were assessed; it is specific and focused on the practice of healthcare waste segregation, which is a crucial component for the rest of waste management. As a limitation, we did not estimate the waste generation rate in each hospital and did not investigate healthcare waste related infections and injuries among health professionals.

## 5. Conclusion

In this study, the practice of healthcare professionals on healthcare waste segregation was poor. In this study, hospital ownership, weekly working hours, knowledge of HCW segregation, HCWM training, the presence of guidelines, SOPs, or instructive posters on HCW segregation, and the availability of color-coded waste bins around the work area were significantly associated with healthcare waste segregation practice.

Therefore, it is highly recommended that hospitals should have ongoing monitoring and assessment of healthcare waste management methods, and providing instructive posters as a tool to promote effective segregation training and making available color-coded bins should be essential to raise awareness of the best handling and management procedures for healthcare waste.

## Figures and Tables

**Table 1:** Sociodemographic characteristics of the respondents in hospitals, Dire Dawa, Eastern Ethiopia.

Variables	Responses	Frequency	Percent
*Age*	<29 years	88	31.4
	30–39	140	50.0
	40–49	41	14.6
	>50 years	11	3.9
*Sex*	Female	173	61.8
	Male	107	38.2
*Marital status*	Divorced	5	1.8
	Married	200	71.4
	Single	72	25.7
	Widowed	3	1.1
*Profession*	Medical doctor	38	13.6
	Health officer	7	2.5
	Laboratory	25	8.9
	Midwifery	26	9.3
	Nurse	184	65.7
*Educational status*	Degree	250	89.3
	Diploma	23	8.2
	Master	3	1.1
	Others	4	1.4
*Work experience*	<2 years	25	8.9
	2–5 years	77	27.5
	5–10 years	87	31.1
	>10 years	91	32.5

The article "Healthcare Waste Segregation Practice and Associated Factors among Healthcare Professionals Working in Public and Private Hospitals, Dire Dawa, Eastern Ethiopia" was published in 2023. Journal: J Environ Public Health.

**Table 2:** Knowledge of health professionals regarding healthcare waste segregation in hospitals in Dire Dawa, Eastern Ethiopia.

Questions	Response	Frequency	Percentage
Do you know about waste segregation?	Yes	264	94.3
	No	16	5.7
Do you know about infectious medical waste?	Yes	269	96.1
	No	11	3.9
Do you know where to put infectious waste in the color-coded bins?	Yes	265	94.6
	No	15	5.4
Do you know where to put sharps and needles?	Yes	271	96.8
	No	15	5.4
Do you know how medical waste is managed?	Yes	259	92.5
	No	21	7.5
Do you know about safety manual at the workplace?	Yes	224	80
	No	56	20
Do you know about the consequence of waste segregation practice?	Yes	234	83.6
	No	45	16.1
Does wearing PPE reduce the risk of infection?	Yes	249	88.9
	No	31	11.1

**Table 3:** Results of factors associated with HCWs segregation practice among healthcare professionals in hospitals, Dire Dawa, Ethiopia.

Variables and responses		*HCWs segregation practices*		COR(95%CI)	AOR(95%CI)
		Good	Poor		
Ownership of hospitals	Public	127	101	0.41 (0.22–0.74)	0.09 (0.03–0.24)^*∗∗*^
	Private	15	37	1	1
Weekly working hours	≤40 hrs	106	85	2.99 (1.78–5.04)	4.28 (2.11–8.68)^*∗*^
	>40 hrs.	39	50	1	1
Knowledge about infectious waste segregation	Adequate	109	80	1.31 (0.97–1.74)	2.42 (1.27–4.61)^*∗∗*^
	Inadequate	36	55	1	1
Ever taken training in HCWM	Yes	56	21	4.61 (2.46–8.63)	2.740 (1.150–6.527)^*∗*^
	No	89	114	1	1
Presence of guideline, SOP, or instructive poster on HCW segregation	Yes	113	53	6.95 (4.08–11.83)	8.21 (3.84–17.54)^*∗*^
	No	32	82	1	1
Availability of color-coded waste bins	Yes	104	77	17.00 (9.06–31.90)	9.53 (4.52–20.10)^*∗*^
	No	41	58	1	1

^*∗*^ *p* value ≤0.05 and ^*∗∗*^*p* value ≤0.001.

## Data Availability

The data used to support the findings of this study are available from the corresponding author upon request.
